This article has been retracted.

# Cytomegalovirus and Herpes Simplex Virus Effect on the Prognosis of Mechanically Ventilated Patients Suspected to Have Ventilator-Associated Pneumonia

**DOI:** 10.1371/journal.pone.0051340

**Published:** 2012-12-07

**Authors:** Yannael Coisel, Sabri Bousbia, Jean-Marie Forel, Sami Hraiech, Bernard Lascola, Antoine Roch, Christine Zandotti, Matthieu Million, Samir Jaber, Didier Raoult, Laurent Papazian

**Affiliations:** 1 Service d’Anesthésie-Réanimation Saint Eloi, Centre Hospitalier Universitaire, and INSERM Unité 1046, Université Montpellier 1, Montpellier, France; 2 UMR CNRS 7278, Université Aix-Marseille, Marseille, France; 3 Réanimation des Détresses Respiratoires et Infections Sévères, Hôpital Nord, Assistance Publique des Hôpitaux de Marseille, and UMR CNRS 7278, Université Aix-Marseille, Marseille, France; University Hospital San Giovanni Battista di Torino, Italy

## Abstract

**Objective:**

Cytomegalovirus (CMV) and herpes simplex virus (HSV) are common viruses that can affect critically ill patients who are not immunocompromised. The aim of this study was to determine whether the identification of CMV and/or HSV in mechanically ventilated critically ill patients suspected of having pneumonia was associated with an increased mortality.

**Design:**

Prospective epidemiological study.

**Setting:**

Medical intensive care unit of a tertiary medical center.

**Patients:**

Ninety-three patients with suspected pneumonia.

**Interventions:**

Patients with suspected pneumonia had bronchoalveolar lavage and blood samples taken to confirm the diagnosis. Antigenemia was used to detect CMV in the blood. Bronchoalveolar lavage samples were submitted to testing using quantitative real-time Polymerase Chain Reaction.

**Measurements and Main Results:**

We identified 22 patients with a CMV infection, 26 patients with an HSV infection and 45 patients without CMV or HSV infection (control group). Mortality at day 60 was higher in patients with a CMV infection than in patients from the control group (55% *vs.* 20%, *P*<0.01). Mortality at day 60 was not significantly increased in the group with HSV infection. Duration of ICU stay and ICU mortality were significantly higher in patients with CMV infections when compared to patients from the control group, whereas ventilator free days were significantly lower in patients with CMV infections when compared to patients from the control group.

**Conclusions:**

In critically ill patients, a CMV infection is associated with an increased mortality. Further interventional studies are needed to evaluate whether treatment could improve the prognosis.

## Introduction

It has been shown for some time that cytomegalovirus (CMV) and herpes simplex virus (HSV) can cause severe disease in immunocompromised patients, either via reactivation of a latent viral infection (the most frequent cause) or via the acquisition of a primary viral infection [1]. More recently, CMV and HSV have been recognized as being pathogenic in critically ill patients who are not receiving immunosuppressive agents [2], [3], [4], [5], [6], [7], [8], [9], [10], [11], [12], [13], [14], [15], [16]. However, the impact of a CMV or an HSV infection on outcome is still debated [2], [10], [13], [14], [17], [18], [19], [20], [21], [22], [23], [24]. Only a few studies have concomitantly evaluated the impact of CMV and HSV on prognosis [2], [7], [12]. In a recent retrospective cohort study of intensive care unit (ICU) patients, Miggins et al. [7] reported that an increased risk of death was associated with several viral species, including CMV and HSV. In a previously published study [2], no such impact on outcome was found for HSV infections. Moreover, the recent use of real-time PCR may have modified the epidemiology of such infections [8], [25]. We hypothesized that the identification of CMV in blood and/or bronchoalveolar lavage (BAL) samples could be associated with a higher mortality rate when compared to controls that do not develop a viral infection. The aim of the present study was therefore to prospectively evaluate the impact that CMV or HSV has on outcome. A control population of patients not developing these viral infections was used as a comparison. This study was performed in a cohort of mechanically ventilated ICU patients that were suspected of having pneumonia.

**Table 1:** Characteristics of patients upon admission to the ICU.

	Overall Population	HSV infection group	CMV infection group	Control group	*p*
	(n = 93)	(n = 26)	(n = 22)	(n = 45)	
**Age (yr), median [IQR]**	63[52–73]	64[54–73]	69[61–75]*	59[43–69]	0.024
**Male gender, n (%)**	55 (59)	14 (54)	14 (64)	27 (60)	0.78
**SAPS II, median [IQR]**	45 [31–55]	50[36–58]	40[31–53]	44[31–55]	0.43
**Direct admission from the community, n (%)**	65 (69)	19 (73)	10 (45)	36 (80)	0.43
**Reason for ICU admission**					
*** Acute respiratory failure***	40 (43)	9 (34)	13 (59)	18 (40)	0.36
*** Acute exacerbation of chronic respiratory insufficiency***	11 (12)	3 (12)	4 (18)	4 (9)	
*** Neurologic failure***	11 (12)	3 (12)	0 (0)	8 (18)	
*** Septic shock***	9 (10)	4 (15)	1 (5)	4 (9)	
*** Postoperative respiratory failure***	8 (8)	1 (4)	2 (9)	5 (11)	
*** Cardiogenic shock***	4 (4)	1 (4)	1 (5)	2 (4)	
*** Hemorrhagic shock***	2 (2)	2 (8)	0 (0)	0 (0)	
*** Miscellaneous***	8 (9)	3 (12)	1 (5)	4 (9)	
**Immunosuppression on ICU admission, n (%)**					
*** No immunosupression***	84 (90)	23 (88)	21 (95)	40 (89)	0.46
*** Chemotherapy***	2 (2)	0 (0)	1 (5)	1 (2)	
*** Long-term corticosteroids***	6 (7)	2 (8)	0 (0)	4 (9)	
*** HIV***	1 (1)	1 (4)	0 (0)	0 (0)	
**Prior ARDS, n (%)**	27 (29)	8 (31)	10 (46)	9 (20)	0.10

SAPS II, simplified acute physiologic score II; ARDS, acute respiratory distress syndrome;

* *p*<0.05 *vs.* No HSV – No CMV.

**Table 2:** Characteristics of patients at the time of diagnosis.

	All	HSV infection group	CMV infection group	Control group	*p*
	(n = 93)	(n = 26)	(n = 22)	(n = 45)	
**Duration of mechanical ventilation prior to suspicion of pneumonia (days), median [IQR]**	2 [2]–[10]	8 [2]–[12] *	7 [2]–[14] *	2 [2]–[5]	0.004
**CPIS score, median [IQR]**	4 [3]–[5]	4 [3]–[5]	3 [2]–[5]	4 [3]–[5]	0.57
**SOFA score (total), median [IQR]**	7 [5]–[9]	6 [3]–[9]	7 [5]–[9]	8 [6]–[10]	0.43
**Prior antibiotics, n (%)**	46 (50)	13 (50)	8 (36)	25 (56)	0.34
**Enteral nutrition, n (%)**	47 (51)	15 (58)	13 (59)	19 (42)	0.30
**Closed-suction system, n (%)**	29 (31)	7 (27)	8 (36)	14 (31)	0.78
**Nasogastric tube, n (%)**	66 (71)	20 (77)	16 (73)	30 (67)	0.64
**Sedation, n (%)**	76 (82)	23 (89)	20 (91)	33 (73)	0.13
**NMBA, n (%)**	26 (28)	8 (31)	8 (36)	10 (22)	0.45
**Anti H2, n (%)**	0 (0)	0 (0)	0 (0)	0 (0)	1
**Sucralfate, n (%)**	1 (1)	0 (0)	0 (0)	1 (2)	0.58
**Antacids, n (%)**	1 (1)	1 (4)	0 (0)	0 (0)	0.27
**Proton-pump inhibitors, n (%)**	84 (90)	24 (92)	19 (86)	41 (91)	0.76
**Statin, n (%)**	9 (10)	2 (8)	4 (18)	3 (7)	0.30
**Strict glycemic control, n (%)**	10 (10)	4 (15)	2 (9)	4 (9)	0.67
**Massive blood transfusion, n (%)**	14 (15)	4 (15)	6 (27)	4 (9)	0.14
**Intrahospital transfer, n (%)**	57 (61)	17 (65)	13 (59)	27 (60)	0.88
**Corticosteroids for septic shock, n (%)**	37 (40)	12 (46)	12 (55)	13 (29)	0.10
**Corticosteroids for ARDS, n (%)**	8 (9)	1 (4)	3 (14)	4 (9)	0.48
**Activated protein C, n (%)**	2 (2)	1 (4)	0 (0)	1 (2)	0.66
**Reintubation, n (%)**	14 (15)	5 (19)	5 (23)	4 (9)	0.26

CPIS, clinical pulmonary infection score; SOFA, sequential organ failure assessment score; NMBA, Neuromuscular blocking agents; massive blood transfusion, replacement of a patient’s total blood volume in less than 24 hours;

* *p*<0.05 *vs.* No HSV – No CMV.

## Materials and Methods

### A. Ethics Statement

The study was approved by the Local Ethics Committee of the Université de la Méditerranée (Marseille, France; approval n° 07-026) which waived the need for written consent, because the protocol did not impact on patient management and complied with standard care in our unit. However, all patients and/or next of kin were informed.

### B. Study Setting and Population

This prospective study was performed in the medical ICU of Sainte-Marguerite University Hospital in Marseille, France. Over a one-year period, all consecutive patients (18 years or older) were prospectively included if they were mechanically ventilated and suspected of having pneumonia. None of the patients were included in a recently published study from the same group [23].

Suspicion of pneumonia was based on the appearance of a new pulmonary infiltrate on chest radiographs, associated with at least 2 of the following criteria: fever >38°C or hypothermia <36°C; white blood cell count >10×10^9^/L or <4×10^9^/L; purulent tracheal secretions; or a decrease in the PaO_2_/FiO_2_ ratio [26], [27].

Fiberoptic bronchoscopy examination was performed in each patient within the first 12 h of suspecting pneumonia. Bronchoalveolar lavage was performed as previously described [27]. BAL samples were tested by RT-PCR, and standard cultures were performed to identify the bacteria and fungi present in the blood and BAL samples [28].

**Figure 1:** Viral load on bronchoalveolar lavage for herpes simplex virus (**Figure 1A**) and cytomegalovirus (**Figure 1B**) according to mortality at day 60.

**Table 3:** Virological results.

	All	HSV infection group	CMV infection group	Control group
	(n = 93)	(n = 26)	(n = 22)	(n = 45)
**HSV status, n(%)**				
*** IgM HSV***	3 (3)	2 (8)	1 (5)	0 (0)
*** IgG HSV***	81 (87)	24 (92)	19 (86)	38 (84)
*** BAL RT-PCR***	31 (33)	25 (96)	6 (27)	0 (0)
**CMV status, n(%)**				
*** IgM CMV***	8 (9)	0 (0)	8 (36)	0 (0)
*** IgG CMV***	72 (77)	18 (69)	20 (91)	34 (76)
*** BAL RT-PCR***	16 (17)	0 (0)	16 (73)	0 (0)
*** Antigenemia***	10 (11)	0 (0)	10 (46)	0 (0)

BAL, bronchoalveolar lavage; RT-PCR, real time polymerase chain reaction.

**Table 4:** Outcomes.

	All	HSV infection group	CMV infection group	Control group	*p*
	(n = 93)	(n = 26)	(n = 22)	(n = 45)	
**Mortality at day 60, n (%)**	32 (34)	11 (42)	12 (55)*	9 (20)	0.012
**ICU Mortality, n (%)**	32 (34)	11 (42)	12 (55)*	9 (20)	0.012
**Duration of mechanical ventilation (days), median [IQR]**	14 [7]–[29]	14.5 [10]–[26]	19.5 [13]–[44] †	10 [3]–[25]	0.009
**VFD at day 28 (days), median [IQR]**	5 [0–22]	5.5 [0–23]	0 [0–0]†	18 [0–26]	0.001
**VFD at day 60 (days), median [IQR]**	37 [0–54]	36.5 [0–55]	0 [0–25]†	50 [11.5–58]	0.001
**Duration of ICU stay (days), median [IQR]**	16 [9]–[30]	18 [11]–[30]	25.5 [15]–[43] †	13 [7–28.5]	0.037
**Shock, n (%)**	40 (43)	10 (39)	17 (77)* ‡	13 (30)	0.001
**Acute renal failure, n (%)**	24 (26)	6 (23)	11 (50)*	7 (16)	0.01
**Bacteremia, n (%)**	19 (20)	3 (12)	10 (46)*	6 (13)	0.004
**ARDS, n (%)**	18 (19)	5 (19)	6 (27)	7 (16)	0.52
**Bacterial VAP, n (%)**	12 (13)	2 (8)	4 (18)	6 (13)	0.55

ICU, intensive care unit; ARDS, acute respiratory distress syndrome; VAP, ventilator-associated pneumonia; BAL, bronchoalveolar lavage; VFD, ventilator-free days.

* *p*<0.01 *vs.* the No HSV – No CMV group;

† *p*<0.05 *vs.* the No HSV – No CMV group;

‡ *p*<0.016 *vs.* the HSV group.

### C. Diagnosis of Pneumonia

One of the investigators made daily rounds in the ICU to identify eligible patients, to determine the onset of pneumonia based on the diagnostic criteria described below, and to record relevant data from the medical records (bedside flow sheets) and the hospital’s mainframe computer, which housed microbiological test results. All chest radiographs were analyzed prospectively by at least two of the investigators.

Confirming a diagnosis of bacterial pneumonia required a suspicion of pneumonia and a BAL quantitative culture that grew at least one microorganism at a concentration ≥10^4^ colony-forming units (cfu)/mL.

### D. Baseline Assessment and Data Collection

Each patient’s hospital chart was prospectively implemented, and the following data were recorded during admission to the ICU: age, sex, Simplified Acute Physiologic Score II (SAPS II) [29], presence of co-morbidities, and presence of previous immunosuppression or previous Acute Respiratory Distress Syndrome (ARDS).

In addition, on the day of sampling, we recorded the Sepsis-related Organ Failure Assessment (SOFA) score [30], the time spent on a mechanical ventilator from admission to the suspicion of pneumonia, and the CPIS score (Clinical Pulmonary Infection Score) modified by Luna [31]. Other relevant clinical characteristics and outcomes complicating the ICU stay following inclusion (ARDS, bacteremia, bacterial ventilator-associated pneumonia (VAP), acute renal failure, shock, ventilator free days and mortality) were also recorded throughout the ICU stay.

**Figure 2:** Meta-analyse of the mortality associated with Cytomegalovirus (CMV) Diagnosis methods are detailed in **table 5**.

**Figure 3:** Meta-analyse of the mortality associated with Herpes Simplex Virus (HSV) Diagnosis methods are detailed in **table 6**.

**Table 5:** Diagnosis Methods used to diagnose CMV infection.

CMV	Sample	Diagnosis methods
Domart 1990 [39]	Blood, urine	Viral culture
Cook 1998 [35]	Lower respiratory tract, tracheal aspiration, blood, skin	Viral culture
Kutza 1998 [37]	Blood	PP65 antigenemia, PCR
Heininger 2001 [4]	Blood, lower respiratory tract	Viral culture, PCR
Cook 2003 [2]	Blood, tracheal aspiration	Serology, viral culture
Jaber 2005 [14]	Blood	PP65 antigenemia
Limaye 2008 [13]	Blood	PCR
Von Muller 2006 [47]	Blood, tracheal aspiration, urine	Serology, PP65 antigenemia, viral culture in blood, tracheal aspiration and urine
Ziemann 2008 [24]	Blood	PCR
Chiche 2009 [23]	Blood, lower respiratory tract	Serology, PP65 antigenemia, viral culture in BAL
Chilet 2010 [34]	Blood, tracheal aspiration	PCR
Heininger 2011 [17]	Blood, tracheal aspiration	PCR
Coisel 2012	Blood, lower respiratory tract	Serology, BAL-PCR, PP65 antigenemia

BAL, bronchoalveolar lavage; PCR, polymerase chain reaction.

**Table 6:** Diagnosis Methods used to diagnose HSV infection.

HSV	Sample	Diagnosis methods
Cook 1998 [35]	Lower respiratory tract, tracheal aspiration, blood, skin	viral culture
Bruynseels 2003 [9]	Lower respiratory tract, throat	viral culture
Cook 2003 [2]	Tracheal aspiration	viral culture
Ong 2004 [38]	Lower respiratory tract, throat	PCR
Engelmann 2007 [36]	Lower respiratory tract, tracheal aspiration, throat	PCR, viral culture, direct immunofluorescence
Luyt 2007 [10]	Lower respiratory tract, tracheal aspiration, bronchial biopsies	BAL-PCR, BAL-viral culture, cytology
Linssen 2008 [18]	Lower respiratory tract	PCR
De Vos 2009 [8]	Lower respiratory tract	PCR
Scheithauer 2010 [19]	Lower respiratory tract, tracheal aspiration	PCR
Smith 2010 [12]	Tracheal aspiration	PCR
Bouza 2011 [48]	Lower respiratory tract	viral culture
Coisel 2012	Blood, lower respiratory Tract	Serology, BAL-PCR

BAL, bronchoalveolar lavage; PCR, polymerase chain reaction.

### E. Serologies and Antigenemia

Viral serology (IgM and IgG) for cytomegalovirus (CMV) and herpes simplex (HSV) were performed using conventional serological methods with an enzyme linked immunosorbent assay (ELISA). Antigenemia for cytomegalovirus was evaluated using a CINA complete kit (Argene SA, Verniolle, France). Briefly, erythrocytes were lysed by mixing 2 mL of EDTA blood with 8 mL of erythrocyte lysing solution and then centrifuged at 300×g for 10 min. Erythrocyte lysis and centrifugation was repeated twice. Then, the supernatant was discarded and the leukocyte pellet was resuspended in 1 mL of phosphate buffered saline (PBS), counted, and then diluted to 2×10^6^ cells/mL. One hundred µL (200,000 cells) were cytocentrifuged at 900 rpm for 3 min on glass slides and air-dried. The slides were fixed with a paraformaldehyde solution for 10 min and washed 3 times with PBS. The cells were then incubated for 30 min at 37°C with a mixture of two monoclonal antibodies (1C3 and AYM). After washing with PBS, the slides were incubated for 30 min at 37°C with a secondary antibody conjugated with fluorescein. The slides were then subjected to 3 final washes with PBS, and examined under a fluorescent microscope. The results are given as the number of positive cells per 200,000 cells. Blood PCR was not routinely done when the study was designed.

### F. Identification of CMV and HSV by PCR on BAL

The presence of CMV and HSV was tested with a quantitative real-time PCR. Viral nucleic acids were extracted from 200 µL of BAL fluids with a MDX workstation using a QIAamp Virus BioRobotMDx Kit (Qiagen, Courtaboeuf, France), as recommended by the manufacturer’s instructions. Quantitative real time PCR for CMV and HSV was performed using a LightCycler® instrument (Roche Diagnostics, Meylan, France) with the QuantiTect Probe PCR Kit (Qiagen). HSV was tested with the PolF (5′-GGGCCAGGCGCTTGTTGGTGTA-3′) and the PolR (5′-CATCACCGACCCGGAGAGGGAC-3′) primer set (Eurogentec, Seraing, Belgium), and the specific TaqMan probe (6FAM-CCGCCGAACTGAGCAGACACCCGCGC-TAMRA) (Applied Biosystems, Courtaboeuf, France). The presence of CMV was tested with the pp65F (5′- GCAGCCACGGGATCGTACT -3′) and the pp65R (5′-GGCTTTTACCTCACACGAGCATT-3′) primer set, and the specific TaqMan probe (6FAM-CGCGAGACCGTGGAACTGCG-TAMRA). The reaction was carried out in 20 µL, in a final volume containing 10 µL of QuantiTect master mix, 0.2 µM of probe, 0.2 mM of each primer, and 4 µL of DNA. The qPCR was initiated by an enzyme-activation incubation at 95°C for 15 min to activate DNA Polymerase, followed by 40 cycles of denaturation at 95°C for 10 s and an annealing-extension step at 60°C for 1 min. Serial dilutions, ranging from 10^2^ to 10^5^ copies/mL, of synthesized sequences that correspond to the targeted viral genes, were used as positive controls. These dilutions were also used to determine the viral load in positive BAL fluids. A CMV and HSV negative specimen was used as a negative control.

### G. Definitions

The **CMV infection group** was defined as patients suspected of having pneumonia with positive CMV DNA detection in BAL fluid and/or positive antigenemia and/or the presence of IgM for CMV. We did not differentiate between endogenous reactivation or exogenous infection as the cause of the active infection. The **HSV infection group** was defined as patients suspected of having pneumonia associated with positive HSV DNA detection in BAL fluid, or the presence of IgM for HSV in patients without CMV identification by antigenemia, real-time PCR or specific IgM. The **“control group”** was defined by the absence of a CMV or HSV infection in patients suspected of having pneumonia.

A bacterial coinfection required the presence of at least one bacteria at a concentration exceeding 10^4^ cfu/mL in the BAL fluid.

### H. Study Outcomes

#### 1. Primary outcome

The primary outcome was mortality for both viruses, evaluated at day 60.

#### 2. Secondary outcomes

Secondary outcomes were the ICU mortality, the day-28 mortality, the number of days with mechanical ventilation, the number of ventilator-free days (days alive and with a successful weaning from mechanical ventilation for at least 48 hrs) between day 1 and day 28, and between day 1 and day 60 [32].

### I. Statistical Analysis

Data are expressed as the median with an interquartile range (IQR) or as number of events (percentage). Continuous variables were compared using a Kruskall-Wallis one-way analysis of variance on ranks, with a pairwise multiple comparisons procedure using Dunn’s method. The chi-squared test was used to compare categorical variables. All reported *P* values are two-sided. For all statistical tests used, a *p* value of <0.05 was considered significant. A Bonferroni method was applied for multiple comparisons when necessary (leading to a significant *p* value of <0.016 when applied). Multiple logistic regressions were used to adjust the day 60 mortality regarding 2 pre-defined variables (SAPS II score on admission and SOFA score the day of BAL).

## Results

### A. Patients Characteristics

#### 1. All patients

During the study period, ninety-three consecutive patients met the inclusion criteria and were prospectively included in the study. Less than one third of all patients were ventilated for ARDS. Ten percent of all patients were previously immunosuppressed (Table 1).

#### 2. Virological status

Twenty-six patients (28%) were included in the HSV group, 22 (24%) in the CMV group, and 45 patients (48%) were negative for both HSV and CMV (control group). Patients from the CMV group were older (Table 1). As shown in Table 2, there was no significant difference between the three groups at the time of diagnosis, excepting a longer duration of mechanical ventilation in patients from the CMV and the HSV groups before the realization of the BAL as compared with the control group.

#### 3. Virological diagnosis

Eighty-one patients (87%) had IgG for HSV and 72 patients (77%) had IgG for CMV. Thirty-one patients had a positive BAL for HSV using RT-PCR (from 6.2×10^3^ to 9.4×10^9^ copies/mL, figure 1A) and 16 patients had a positive BAL for CMV using RT-PCR (from 9.9×10^3^ to 3.1×10^7^ copies/mL, figure 1B). Table 3 shows that antigenemia and RT-PCR were positive for 46% and 73% of the patients exhibiting an active CMV infection, respectively. Eight of the patients with a positive antigenemia for CMV also had a positive RT-PCR for CMV. Finally, all but four patients from the CMV infection group had a positive RT-PCR for CMV performed on BAL samples and/or a positive antigenemia. Only one patient from the HSV group presented IgM with a negative RT-PCR for HSV on BAL. Six patients from the CMV group also had a positive RT-PCR for HSV. By definition, no patient from the HSV group had a positive antigenemia or RT-PCR for CMV.

A concomitant confirmed bacterial lung infection was present in 11 patients from the HSV group (42%), 11 (50%) from the CMV group and 16 (36%) from the control group (*p* = 0.52). Gram-negative bacilli represented respectively 79%, 62% and 72% of the bacteria cultured from BAL.

### B. Outcomes (Table 4)

Mortality at day 60 was higher in patients with a CMV and/or a HSV infection [48% (CI 95 from 35% to 62%)] compared to patients from the control group [20% (CI from 11% to 34%)] (*p*<0.005). More specifically, mortality at day 60 was higher in patients with a CMV infection [55% (CI 95 from 35% to 73%)] compared with control patients [20% (CI from 11% to 34%)] (*p*<0.01). This difference remained significant after adjusting for age, SAPS II score on admission and SOFA score on the day of diagnosis. Mortality at day 60 was not significantly higher in the HSV group [42% (CI from 26% to 61%)] compared to the control group. As shown in Figure 1, there was no relationship between mortality at day 60 and the viral load for both the CMV group and the HSV group.

Ventilator-free days at D28 and D60 were significantly lower in patients developing an active CMV infection than in patients from the control group. The duration of ICU stay and the ICU mortality rate were significantly higher in patients developing an active CMV infection than in patients from the control group (Table 4). However, there was no difference between the CMV group and the HSV group regarding these parameters. There was no correlation between the viral load and the number of ventilator-free days at D28 and D60 (data not shown).

Complications such as bacteremia, acute renal failure or shock were significantly more frequent in the CMV group (Table 4). In contrast, there were no increases in the rate of bacterial VAP or ARDS following virus identification in the CMV group when compared to the other two groups.

## Discussion

The present study suggests that an active CMV infection in critically ill patients increases both crude and adjusted mortalities at day 60. CMV infection was also associated with less ventilator free days at day 28 and day 60, and an increased duration of ICU stay compared with patients without CMV and HSV identification.

Infection with a *Herpesviridae* family virus, namely CMV and HSV, is very common in the general population, whether they are immunosuppressed or not [33], [34], [35], [36], [37], [38]. In critically ill patients, the incidence of both active CMV and HSV infection is matter of controversy [14], [23]. Moreover, many studies were performed in trauma or surgical patients. Serological positivity for CMV reported in critically ill patients ranged from 13% [39] to 100% [40]. Respiratory samples positive for CMV ranged from 0% [41] to 13% [4], antigenemia ranged from 0% [42] to 17% [14], and even 85% in one study [23]. However, the use of open lung biopies found that up to 50% of patients with ARDS were infected with CMV [16]. These differences could be explained by different diagnostic methods for the detection of CMV, including viral culture, antigenemia and PCR assays [22]. Previous studies used culture-based assays (low sensitivity and time-consuming), whereas more recent studies have used antigenemia (more sensitive and quantitative results) or PCR assays [13]. Nevertheless, none of these methods have been validated in ICU patients. Moreover, our results should take in account the relative lack of sensitivity and specificity of some of these diagnostic methods (serology for example). It was likely that some patients with positive virus may actually have infection, whereas other with positive samples may just be false positive. The newest diagnostic methods have not been validated in ICU patients. However, in immunocompromised patients, techniques such as PCR and antigenemia present an adequate diagnostic accuracy [43], [44].

CMV reactivation in intensive care patients is not trivial. Indeed, in a study using a murine model, Cook et al. showed that CMV reactivation caused abnormal tumor necrosis factor-α expression and induced abnormal pulmonary fibrosis, both of which were prevented with ganciclovir [45]. Reactivation of CMV could lead to an increased duration of ventilation or ICU stay in non-immunosuppressed patients in an intensive care setting [2], [14], [23], [24], [46], [47]. A human study found an independent correlation between CMV reactivation and morbidity in non-immunosuppressed patients [17], however, there was no correlation with mortality. Another human study found a significant increased mortality rate in patients expressing CMV, but could not demonstrate a cause-effect relationship [20]. In our study, we could identify factors associated with positive CMV samples, but causative links between both had not been addressed.

To our knowledge, this is the first study indicating that an active CMV infection in critical care patients increased crude and adjusted mortality at day 60. Our results are concordant with those of Heininger et al. [4], who found that the mortality rate tended to be higher in patients with active CMV infections, with a significant increase in ICU length of stay in survivors. Limaye [13] also found and association between CMV reactivation and a composite end point (prolonged hospitalization or death). In our unit, all patients with an active CMV infection were treated with gancyclovir, which make it difficult to conclude regarding the efficacy of this treatment. Only an interventional trial could conclude if CMV is definitely responsible for a longer duration of mechanical ventilation/LOS. Indeed, a longer duration of exposure to mechanical ventilation could be associated with an increased risk to identify CMV without any impact on prognosis. This is unlikely because in the present study, patients from the control group were ventilated invasively for a longer period than the time to identify CMV in the CMV group.

Figures 2 and 3 represent two meta-analyses of the mortalities associated with CMV and HSV. Even if the diagnostic criteria and the studied populations are very different from one study to another (Tables 5 and 6), these analyses suggest that both CMV and HSV are associated with increased mortality rates.

This study strongly suggests that CMV reactivation in critically ill patients is associated with increased mortality. With respect to HSV infections, its impact on various outcome measures seems to be less important when compared to patients infected with CMV. However, only a trial evaluating the efficacy of an anti-viral treatment in ICU patients could demonstrate that CMV and/or HSV alter outcome.
